# Psoriasis Vulgaris of Blood Heat Syndrome in Plasma Based on Widely Targeted Techniques

**DOI:** 10.1155/2022/2113769

**Published:** 2022-04-15

**Authors:** Xueyong Tang, Juan Gong, Yourang Jiang, Xi Chen, Dongwei Qi, Xin Li

**Affiliations:** ^1^Department of Dermatology, Chongqing Hospital of Traditional Chinese Medicine, Chongqing 400021, China; ^2^Hunan University of Chinese Medicine, Changsha 410208, China

## Abstract

Traditional Chinese medicine classifies psoriasis (Ps) according to clinical manifestations, and its different clinical manifestations imply the pathogenesis and material evolution basis of Ps, especially biomarkers that are meaningful to identification of Ps, treatment response, and elucidation of the pathogenesis of the disease. This study aims to screen differential metabolites in plasma of psoriasis vulgaris (PV) of blood heat syndrome based on a widely targeted metabolomic technique and to analyze syndrome metabolic markers and metabolic pathways. Forty-five PV patients were recruited, including 21 cases of the blood heat syndrome group (BH-PPG), 24 cases of the non-blood-heat syndrome group (NBH-PPG), and 30 healthy cases of the normal control group (NPG). The UPLC-MS/MS detection platform, a self-developed database, and multivariate statistical analysis were applied to investigate the plasma metabolic differences. The biomarkers related to blood heat syndrome were screened using the principal component analysis method. A total of 479 metabolites were detected in the three groups of plasma samples; 72 different metabolites were sorted out in the BH-PPG/NPG group, 82 in the NBH-PPG/NPG group, and 8 in the BH-PPG/NBH-PPG group. Differential metabolites mainly consist of metabolites of organic acids, amino acids, carbohydrates, and nucleotides. Multiple metabolites ginkgolic acid, pyrroloquinoline quinone, L-aspartic acid, and citramalic acid were expected to be the potential biomarkers of blood heat syndrome PV. The formation and evolution processes may be associated with disorders and regulation of metabolic pathways, ferroptosis, carbon metabolism, and purine metabolism.

## 1. Introduction

Psoriasis (Ps) is one of the most common chronic recurrent systemic dermatoses clinically [1], with a mounting incidence every year. The global prevalence rate is 0.51%–11.43% [2], and the recent incidence in China is 0.47% [3]. Because the disease has characteristics such as a long course, high recurrence rate, and low cure rate, it seriously impacts the physical and mental health of patients. Traditional Chinese medicine has unique advantages in the recognition and differentiation of this disease. Based on literature research and expert consensus, the clinical differentiation of psoriasis vulgaris (PV) presents three basic syndromes: blood heat syndrome, blood stasis syndrome, and blood dryness syndrome [4]. Zhao Bingnan was the first to put forward the basic pathogenesis of Ps that “there is long-term accumulated internal heat and stagnation of blood.” Blood heat syndrome is the most important syndrome type in the progressive stage. It is not only the beginning of the onset but also essential to the transformation of the disease and syndrome [5]. However, the complexity of its pathogenesis, the internal reality and external deficiency of the syndrome, the multidimensional interface, the nonlinearity, and the formation and evolution of the syndrome need to be further clarified.

As the basic research of traditional Chinese medicine (TCM) syndromes and treatment on clinical metabolomics advances gradually, its advantages of multilevel, multitarget, and overall dynamics and temporal and spatial complexity have provided an effective solution for the investigation of the material basis and biomarker research of TCM syndromes [6]. In recent years, based on the metabolomics technique and bioinformatics methods, certain achievements have been made in research on the basis of Ps TCM syndromes and the efficacy evaluation of prescriptions [7]. However, the techniques of magnetic resonance imaging and nontargeted metabonomics methods, which have been mostly used, provide relatively low sensitivity and quantitative accuracy. Lately, the widely targeted metabolomics integrates the advantages of targeted and nontargeted ones, which is more applicable for the detection of low-to-medium abundant metabolites [8, 9]. Moreover, psoriasis vulgaris of blood-heat syndrome was diagnosed through different symptoms from the non-blood-heat syndrome [10]. It is assumed that differential metabolites are found between psoriasis vulgaris of blood-heat syndrome and non-blood-heat syndrome based on widely targeted metabolomics. The present study applies a widely targeted metabolomics approach and screens out differential metabolites and metabolic pathways in plasma samples of blood heat syndrome PV and intends to explore the material basis and evolution of PV syndrome based on the pathogenesis of blood heat syndrome.

## 2. Materials and Methods

### 2.1. Data Collection

#### 2.1.1. Data Source

The 45 Ps volunteers were patients who visited the dermatology department of Chongqing Traditional Chinese Medicine Hospital (Daomenkou Division) from January to June 2019. There were 21 patients in the blood heat syndrome group (BH-PPG), and non-blood heat syndrome groups (NBH-PPG) included 13 for the blood stasis syndrome group (BS-PPG) and 11 for the blood dryness syndrome group (BD-PPG). There were also 30 volunteers in the normal control group (NPG) who were recruited from the physical examination center of this hospital and determined to be healthy during the same period. This project was approved by the Ethics Committee of Chongqing Traditional Chinese Medicine Hospital. All patients and healthy volunteers provided signed informed consent and volunteered to participate in this project.

#### 2.1.2. Diagnostic Criteria

The western medicine diagnostic criteria for psoriasis vulgaris were referred to guidelines as previously published [11, 12]. Diagnosis of TCM syndromes referred to “Clinical Pathways of Traditional Chinese Medicine” diagnosis criteria of TCM clinical pathway syndromes of psoriasis (psoriasis vulgaris) [12]. Western medicine diagnosis and syndrome differentiation of cases were carried out by TCM researchers of attending physicians or above in the Department of Dermatology of this hospital who had been trained and who strictly implemented the previously described diagnostic criteria.

#### 2.1.3. Inclusion Criteria

The inclusion criteria were as follows: ① patients should conform to the diagnostic criteria of western medicine diagnosis of PV and TCM blood heat syndrome, blood stasis syndrome, and blood dryness syndrome diagnosis of PV. ② Patients were of 18–65 years of age. ③ Patients should have no systemic diseases in the circulation, digestion, and endocrine systems, blood, and connective tissue and no other acute or chronic inflammatory or autoimmune dermal diseases except for Ps. ④ During the period from onset to treatment, no systemic or local medications including immunosuppressive agents, glucocorticoid steroid hormones, retinoids, antihistamines, biological agents, and traditional Chinese medicine should be administered, as well as no acceptance of physical therapy; ⑤ Patients should eat a light diet, take rest regularly, avoid bad habits such as smoking or drinking 6 weeks before onset. ⑥ Subjects are those who volunteered for the project and could enjoy the rights and fulfil the obligations as required. ⑦ Patients should have signed the informed consent.

#### 2.1.4. Exclusion Criteria

Subjects with one or more of the previously described inclusion criteria that could not be met were excluded.

### 2.2. Sample Collection and Treatment

Both patients with PV syndromes and healthy volunteers fasted in the morning before collection of 3 to 5 mL of blood samples, which was carried out using tubes containing an anticoagulant. Immediately after blood collection, the tubes were gently inverted to mix the blood samples evenly 5 to 10 times to ensure the effect of the anticoagulant. The samples, after being collected within 30 min, were centrifuged at 3 000 rpm at 4°C for 10 to 15 min. Subsequently, 100 *μ*L of the supernatant (plasma) was aspirated on ice, transferred to an EP tube, and stored in a refrigerator at −80°C for later use.

### 2.3. UPLC-MS/MS Analysis Conditions

The liquid phase conditions mainly include ① chromatographic column: Waters ACQUITY UPLC HSS T3 C18 1.8 *µ*m, 2.1 mm ∗ 100 mm; ② mobile phase: phase A used ultrapure water (0.04% acetic acid), and phase B was acetonitrile purchased from Merck (0.04% acetic acid); ③ elution gradient: 0 min water/acetonitrile (95 : 5 V/V), 11.0 min 5 : 95 V/V, 12.0 min 5 : 95 V/V, 12.1 min 95 : 5 V/V, and 14.0 min 95 : 5 V/V; ④ flow rate was at 0.4 ml/min, with a column temperature of 40°C and injection volume of 2 *μ*L. The standard reagent was chromatographically pure grade (China, BioBioPha). The experiment was performed on a shim-pack ultra-performance liquid chromatograph (Japan, SHIMADZU) and a QTRAP® 6500 + tandem mass spectrometer (USA, SCIEX). The mass spectrometry conditions mainly included the following: the temperature of the electrospray ionization source (ESI) is 500°C; the mass spectrum voltage is 5 500 V (positive) and −4 500 V (negative); and the pressure of ion source body I (GS I) is 55 psi, ion source body II (GSII) is 60 psi, and curtain gas (CUR) is 25 psi. The parameter of collision-induced ionization (CAD) was configured is high. Each ion pair of the QTRAP system was scanned based on the optimized declustering potential (DP) and collision energy (CE) [13].

### 2.4. Data Analysis

The metware database (MWDB), developed by MetWare Biotechnology Co. Ltd., was adopted for qualitative analysis using the retention time of the detected substance, the information of the precursor-product ion pair, and the secondary spectrum data. After obtaining the metabolite spectrum data of different samples, the characteristic ions of each substance were screened out using the QTRAP system. Analyst 1.6.3 and MultiQuant software were also applied to mass spectrometry quantitative analysis. Meanwhile, the construction of a reliable mathematical model adopted multivariate statistical analysis methods. Principal component analysis (PCA) was initially performed on the samples to observe the variability of the differentiated grouping samples. Based on the metabolite content, the range method was used for normalization, and the R software (https://www.r-project.org/) was applied to perform hierarchical cluster analysis (HCA) on the metabolites of different samples. Then, orthogonal partial least squares discriminant analysis (OPLS-DA) was used to distinguish the overall differences in metabolites between groups. Using the obtained multivariate analysis of the variable importance projection (VIP) of the OPLS-DA model, the metabolites of different species or tissues could be initially screened. Meanwhile, the *p* value or fold change in univariate analysis could be combined to further screen out the metabolites with VIP ≥1, fold change ≥2, or fold change ≤0.5 as significantly different metabolites.

## 3. Results

### 3.1. Clinical Baseline Comparison

The general data and disease conditions of the disease group and the normal control group are shown in Table 1. There are no significant differences in gender, age, and BMI between the control group and the disease group. In addition, there are also no significant differences in family history and BMI between BH-PPG and NBH-PPG, whereas significant differences are revealed in gender, age, course of disease, and psoriasis area severity index (PASI) scores.

### 3.2. Plasma UPLC-MS/MS Inspection Results

#### 3.2.1. Sample Quality Control Analysis

The quality control sample (QC) was prepared by mixing the sample extracts, which was subsequently applied for monitoring the sample repeatability under the same processing method to obtain the trusted Internet connection (TIC) overlay detected by the mass spectrometry (Figure 1). The results indicate that the total ion current curves present a high overlap, detected using the metabolites, and the retention time and peak intensity are consistent, indicating that the signal stability is better when the mass spectrometer detects the same sample at different time points.

#### 3.2.2. PCA and OPLS-DA Results between Groups

Pairwise comparison obtained the three-dimensional PCA structures of BH-PPG v NPG, NBH-PPG v NPG, and BH-PPG v NBH-PPG, and OPLS-DA scores and the S-plot (Figure 2), indicating an apparent trend of separation between groups. The results reveal that there is no crossover and overlap among the groups, with an apparent separation trend, and significant differences in plasma metabolites.

#### 3.2.3. Differential Metabolite Screening Analysis

Based on OPLS-DA results, the metabolites with VIP ≥1, fold change ≥2, or fold change ≤0.5 were selected as significantly differentiated metabolites. Compared with the normal group, BH-PPG has 72 different metabolites, including ginkgolic acid and pyrroloquinoline quinone (Figure 3). They mainly consist of the metabolism of organic acids and their derivatives, followed by the metabolism of amino acids, carbohydrates, nucleotides, and their metabolites. There are 65 overlapped different metabolites with NBH-PPG (Table 2). BH-PPG presents 7 characteristic different metabolites compared with the normal group, including marked upregulation of L-petaminoacetic acid, L-amphetaminoacetic acid, and N-methyl-L-glutamic acid and marked downregulation of acadizine, 2-(methylthio)ethanol, neopterin, benzoic acid, and inositol; There are 17 different metabolites in the NBH-PPG group, including adenosine-3′-phosphate. Comparing the BH-PPG and NBH-PPG groups, four differential metabolites—1-naphthol, cortisol, inosine, and (±) 12-hydroxy-5Z, 8Z, 10E, 14Z-eicosatetraenoic acid—are markedly upregulated, whereas 4 differential metabolites—3,4,5-trimethoxycinnamic acid, 4-pyridoxic acid, mandelic acid, and p-hydroxyphenylacetic acid—are significantly downregulated, as shown in Table 3.

#### 3.2.4. Metabolic Pathway Analysis

The KEGG database [14] was applied to annotate and enrich the selected differential metabolites, which were subsequently classified according to the types of pathways in KEGG (Figures 4 and 5). The results reveal that compared with the normal group, there are 23 entries of metabolic pathways in BH-PPG with differential metabolites ≥4 and 9 entries of metabolic pathways with *p* value ≤0.05 involve metabolic pathways, ABC transporters, antibiotic biosynthesis, carbon metabolism, ferroptosis, purine metabolism, galactose metabolism, glutathione metabolism, and phosphotransferase system (PTS). Among them, metabolic pathway q-values (corrected *p*-values), including ferroptosis (Figure 6) and carbon metabolism (Figure 7), are all less than 1, and the enrichment difference is significant.

## 4. Discussion

TCM diagnosis and treatment of psoriasis give priority to symptom differentiation and cause exploration of disease treatment with the corresponding prescriptions and syndromes. Syndrome is the starting point and the core of syndrome differentiation for disease treatment, and it is the bridge and key to the inheritance of principle, prescription, and medication [15]. The recent research on the standardization and material basis of psoriasis syndrome classification is mainly based on macroanalysis such as big data literature research and expert consensus. Despite that, there is some exploration on the microbiological basis of syndromes, and it is difficult to systematically clarify the formation and evolution mechanism of syndromes under the guidance of reduction theory [16]. Metabonomics starts from the terminal level of the human metabolic network, characterizes the response and regulation of the overall functional state of the body under the influence of pathogenic factors, and reveals essential metabolites closely related to disease and syndrome development. It also explores the formation and evolution of disease and syndrome [17, 18]. Based on a widely targeted metabonomics technique, this study analyzes plasma differential metabolites and screens specific key metabolic biomarkers for the pathogenesis and evolution of PV with blood heat syndrome.

Comparison of general data reveals that the condition is more serious in BH-PPG and the PASI scores are significantly higher than those of the NBH-PPG group. The total course of the disease is slightly short, with more men than women and younger age. These factors indicate that most of the blood-heat syndrome is in a progressive stage, which confirms that blood-heat syndrome is not only the beginning of the onset or recurrence of the disease but also key to the transformation of the disease. Analysis of widely targeted metabolomics shows that there are significant differences in plasma metabolism between BH-PPG, NBH-PPG, and the normal control groups. Comparing the syndrome group with the normal group, 65 overlapped differential metabolites including ginkgolic acid, pyrroloquinoline quinone (PQQ), L-aspartic acid, citramalic acid, and 3-hydroxybutyric acid are identified, and metabolic categories mainly involve organic acids, amino acids, carbohydrates, and nucleotides and its metabolites.

Organic acid is a carboxylic acid in the metabolism of amino acid, lipids, and sugar. It is widely distributed in plants. The human body develops disease due to certain enzyme depletion resulting from the accumulation of related carboxylic acids and their metabolites [19]. In this study, organic acids and their derivatives account for 23.29% of the different metabolite categories. The top 20 organic acids with significant differences include ginkgolic acid, PQQ, arginaminosuccinic acid, Β-hydroxypyruvic acid, methyl isobutyrate, 2-hydroxybutyric acid, and methyl maleic acid. Among them, ginkgolic acid is present mostly in *Ginkgo biloba*. The research on the relationship of ginkgolic acid with diseases is mostly focused on its toxic and side effects such as sensitization, genotoxicity, and hepatorenal cytotoxicity [20, 21]. However, there are few studies on its metabolism in vivo and in vitro, and the apparent increase in plasma ginkgolic acid may be related to some drug oxidative metabolic enzymes. Abnormal expressions of CYP1A1 and CYP2E1, members of the cytochrome P450 (CYP450) family, are closely related to the occurrence and development of psoriasis [22], which may affect the normal metabolism of ginkgolic acid, thereby leading to a marked elevation in plasma expression levels. PQQ can scavenge intracellular oxygen-free radicals and avoid oxidative damage of tissues and cells, and it can repair mitochondrial dysfunction [23]. The marked increase in plasma PQQ expression may be involved in the inflammatory mechanism of Ps by affecting the function of mitochondria. Argininosuccinic acid ornithine is the intermediate product of circulation. As a precursor of arginine, it can be generated by the condensation of citrulline and aspartic acid under the action of argininosuccinate synthase in the liver and kidney. 3-hydroxybutyric acid is intimately correlated to energy metabolism disorders in organisms and diabetes. It can improve tissue damage, metabolic disorders, and protein metabolism as well as induce tumor cell apoptosis [24, 25]. Meanwhile, the downregulation of expression may be involved in the PV onset. The differential metabolism of some organic acids, namely, ginkgolic acid, selected in this study has not been reported in the previous literature, and its effect mechanism in the pathogenesis of PV or the formation of syndromes needs further exploration.

Second, 13 kinds of amino acids and their derivatives citramalic acid, L-aspartic acid, L-glutamic acid, and glutamate account for 19.18% of the differential metabolite categories. As the main place of amino acid metabolism in the human body, the liver plays an important role in the intake, synthesis, and secretion of amino acids. The level of amino acid metabolism directly reflects the state of liver cell metabolism. Studies have shown that patients with advanced psoriasis have abnormal amino acid metabolism and ratio imbalance [26] and liver and kidney amino acid metabolism disorders, so the abnormal expression of amino acid levels in plasma may be involved in the pathogenesis and progression of Ps [27]. This study reveals that the significant up-regulation of L-aspartic acid, L-glutamic acid, and glutamate is consistent with previous research results. The increased expression of aspartic acid and proline might be involved in the protein biosynthesis of Ps and excessive proliferation of keratinocytes [28, 29]. The expression level of glutamate is positively correlated with the severity of Ps lesions [30]. The expression of citramalic acid is markedly down-regulated. As an important node of the tricarboxylic acid (TCA) cycle, abnormal expression will disrupt the metabolism of the TCA cycle, thereby affecting the glycolysis process. These metabolic changes enhance the production of mitochondrial reactive oxygen species and the unfolded protein response, which in turn causes an immunoinflammatory response in psoriasis marked by IL-23 and the onset of this disease [31].

In addition, nucleotides, carbohydrates, and their metabolites are in a higher proportion. Nucleotides are mainly involved in a variety of physiological functions, namely, energy metabolism and coenzyme regulation, the metabolism of which consists of three processes—synthesis, decomposition, and regulation. Some research evidence has indicated that abnormal purine nucleotide metabolism can affect the expression of genes and proteins by regulating signal transduction pathways, and a variety of enzymes involved in its metabolism are closely related to tumor cell proliferation, transformation, invasion, metastasis, and drug resistance [32]. Nucleotide metabolites in the BH-PPG group differ greatly from those of the normal group, including 2-hydroxy-6-aminopurine, guanine, guanosine, inosine, and arabinoinosine, suggesting that abnormal purine nucleotide synthesis and catabolism might be involved in Ps progression. Carbohydrates are the main components and major energy supplying substances of living cell structures, which have an important function of regulating cell activities. The metabolic processes contain sugar catabolism and anabolism. The oxidation and decomposition require multiple vitamins and metal ions as coenzymes. It is, therefore, the deficiency of coenzymes that can cause glucose metabolism disorders. Furthermore, the process is also affected by oxygen uptake, metabolic intermediates, hormones, and neurohumour of the body. The expressions of carbohydrate metabolites D-mannose, *β*-D-glucose, D-sorbitol, and N-acetylglucosamine 1-phosphate are significantly different, suggesting abnormal glucose metabolism in psoriasis with blood-heat syndrome.

Among the nine metabolic pathways with significantly enriched differential metabolites, ferroptosis [33], carbon metabolism [34], and purine metabolism [35] with *q* value < 1 are closely related to Ps pathogenesis. Among them, the ferroptosis metabolic pathway is mainly enriched with differential metabolites of the amino acid, including L-cystine, L-cysteine, reduced glutathione, glutamate, and L-glutamic acid. The carbon metabolism pathway is mainly enriched with *β*-D-glucose, L-cysteine, D-xylulose-5-phosphate, leucovorin, Β-hydroxypyruvic acid, L-glutamic acid, glutamate, and L-aspartic acid. The purine metabolism pathway is mainly enriched with differential metabolites of the nucleotide, including guanine, hypoxanthine, inosine, guanosine, and adenosine. Metabolic pathway analysis indicated that the formation and evolution of psoriasis with blood-heat syndrome may involve a series of complex metabolic disorders and adjustment processes, namely, liver and kidney amino acid metabolism, energy metabolism, and coenzyme regulation related to nucleotides.

In conclusion, this study analyzes plasma metabonomics of PV with blood heat syndrome and screens multiple differential metabolites of ginkgolic acid, PQQ, L-aspartic acid, and citramalic acid. These metabolites are considered to be potential biomarkers of blood-heat syndrome PV. Specific disease and syndrome metabolic pathways contain carbon metabolism, ferroptosis, and purine metabolism. The exploration of these differential metabolites and metabolic pathways can provide indicators for diagnosis and treatment of Ps-based blood-heat pathogenesis. Meanwhile, it also offers a new objective basis for revealing the material basis of the occurrence, development, and outcome of the pathogenesis of blood heat disease. Some potential markers for psoriasis have been identified at the genome, transcriptome, proteome, and metabolome level in previous research. This study not only explores the potential metabolic markers of PV based on the widely targeted metabolomic technique but also investigates the metabolic markers and metabolic pathways of two PV syndromes (blood heat syndrome and non-blood-heat syndrome) identified by TCM. Unfortunately, this study still has several limitations. The uncertainty of the dynamic changes during the metabolic process and the characteristics of multifactor interference of metabolites are the causes of difficulty in the reproducibility of metabolic data for subsequent research teams. Several differential metabolites have not been reported in the previous literature, and their effect mechanism in the pathogenesis or syndrome formation of psoriasis has not been further studied. In addition, despite that metabolic pathways and network analysis present some essential biological information, the clinical applicability of relevant evidence remains to be further explored. In subsequent projects, multisample, multilevel, and in-depth research can be performed using serum, urine, feces, saliva, and injured skin tissues to more comprehensively and accurately explore the mechanism of formation and evolution of the pathogenesis of blood heat PV.

## 5. Conclusions

Here, we analyzed plasma metabonomics of PV with blood heat syndrome and found multiple differential metabolites of ginkgolic acid, PQQ, L-aspartic acid, and citramalic acid, which are considered to be potential biomarkers of blood-heat syndrome PV. It is helpful for western medicine to explore the identification of PV syndrome and the mechanism of disease progress, promote the development of western medicine in the identification of PV blood heat syndrome, and facilitate the progress of the PV diagnosis and treatment method.

## Figures and Tables

**Figure 1:** QC sample TIC overlap detected by mass spectrometry. (a) QC_MS_TIC-N (normal control group) (b) QC_MS_TIC-P (disease group).

**Figure 2:** PCA and OPLS-DA plots of plasma samples in each group. *Note.* A1/B1, A2/B2, and A3/B3 represent the PCA three-dimensional structures, OPLS-DA scores, and S-plot of BH-PPG/NBH-PPG and the normal control group, respectively; C1, C2, and C3 represent the PCA three-dimensional structures, OPLS-DA scores, and S-plot of BH-PPG and NBH-PPG groups, respectively.

**Figure 3:** Differential metabolites' volcano map.

**Figure 4:** KEGG differential enrichment classification chart. Note: the vertical ordinate represents the KEGG metabolic pathways, and the horizontal axis represents the number of metabolites annotated to the pathway and the ratio to the total number of annotated metabolites.

**Figure 5:** KEGG differential enrichment bubble chart. *Note.* The horizontal axis represents the corresponding rich factor of each pathway, and the vertical ordinate represents the pathways. The dot color represented *p* values; the darker the red, the more significant the enrichment. The dot size represents the number of enriched differential metabolites.

**Figure 6:** Ferroptosis metabolic pathway. *Note.* Red indicated markedly up-regulated content of metabolites in the experimental group. Blue indicated no marked change of the metabolite which had been detected. Green indicated markedly down-regulated content of metabolites in the experimental group. Cause for the phenotypic differences among the research subjects was identified through metabolic pathways.

**Figure 7:** Carbon metabolic pathway. *Note.* Red indicated markedly up-regulated content of metabolites in the experimental group. Blue indicated no marked change of the metabolite which had been detected. Green indicated markedly down-regulated content of metabolites in the experimental group. Cause for the phenotypic differences among the research subjects was identified through metabolic pathways.

**Table 1:** General data baseline comparison in each group.

Item	Normal control group (30 cases)	Disease group (45 cases)	Blood heat group (21 cases)	Non-blood heat group (24 cases)	Blood stasis group (13 cases)	Blood dryness group (11 cases)
Gender (male/female)	16/14	24/21	14/7^*∗∗*^	10/14	4/9	6/5
Age (years)	36.90 [19, 56]	41.51 [18, 65]	35.95 [18, 54]^*∗∗*^	46.38 [23, 65]	45.46 [25, 65]	47.45 [23, 65]
BMI index	21.68 [15.68, 25.68]	23.99 [15.57, 32.46]	24.20 [15.57, 32.46]	23.81 [17.96, 28.93]	23.71 [19.52, 28.13]	23.92 [17.96, 28.93]
Family history (yes/no)		18/27	10/11	8/16	3/10	5/6
Course (year)		10.02 [0.3, 30]	7.88 [0.5, 40]^*∗*^	11.90 [0.5, 40]	11.65 [0.5, 36]	12.18 [4, 40]
PASI scores		13.62 [0.6, 28.8]	15.73 [0.6, 28.8]^*∗∗*^	11.78 [1.8, 27.0]	11.41 [1.8, 22.5]	12.21 [2.6, 27.0]

*Note.* Except for gender and family history, the additional data of each item are represented by the median [minimum, maximum]; ^*∗*^*p* < 0.1 and ^*∗∗*^*p* < 0.05.

**Table 2:** Significantly different metabolites of BH-PPG and NBH-PPG from the normal control group.

Index	Differential metabolites	Metabolite categories	BH-PPG v NPG		NBH-PPG v NPG		Type
			VIP value	Log2FC	VIP value	Log2FC	
MEDN636	Ginkgolic acid	Organic acids and the derivatives	2.01	19.59	1.96	19.54	Up
MEDN196	Pyrroloquinoline quinone	Organic acids and the derivatives	2.01	16.57	1.96	16.65	Up
MEDN009	L-Aspartate amino	Amino acids and the metabolites	2.10	14.85	1.96	14.96	Up
MEDN195	Phosphopyridoxal	Pyridine and the derivatives	2.10	11.79	1.95	11.73	Up
MEDN499	Argininosuccinic acid	Organic acids and the derivatives	1.42	4.19	1.37	4.14	Up
MEDP443	Leucovorin	Pteridine and the derivatives	1.83	3.13	1.80	3.18	Up
MEDN506	N-Acetylglucosamine 1-phosphate	Carbohydrate and the metabolites	2.00	3.02	1.92	3.09	Up
MEDP831	DL-1-Amino-2-propanol	Alcohols	1.63	2.35	1.25	2.51	Up
MEDP016	L-Glutamic acid	Amino acids and the metabolites	1.79	1.90	1.61	1.72	Up
MEDP860	Glutamate	Amino acids and the derivatives	1.76	1.80	1.51	1.48	Up
MEDN206	Citromalic acid	Amino acids and the metabolites	2.10	−19.7	1.96	−19.7	Down
MEDN292	3-Hydroxybutyric acid	Organic acids and the derivatives	2.10	−18.98	1.96	−18.98	Down
MEDN244	Orotic acid	Coenzymes and vitamins	2.10	−18.11	1.96	−18.11	Down
MEDN484	Β-Hydroxypyruvic acid	Organic acids and the derivatives	1.96	−18.05	1.83	−18.05	Down
MEDP718	Methyl isobutyrate	Organic acids and the derivatives	2.10	−15.88	1.96	−15.88	Down
MEDN283	2-Hydroxybutyric acid	Organic acids and the derivatives	2.10	−15.81	1.96	−15.81	Down
MEDN726	Capraldehyde	Aldehydes	2.10	−15.03	1.96	−15.03	Down
MEDN738	2, 6-Dimethylnaphthalene	Benzene and the derivatives	2.10	−15.01	1.96	−15.01	Down
MEDP151	2-Hydroxy-6-aminopurine	Nucleotide and the metabolites	2.10	−14.51	1.96	−14.51	Down
MEDN469	Citraconic acid	Organic acids and the derivatives	2.07	−11.55	1.96	−19.11	Down

*Note.* List of top 10 upregulated and downregulated differential metabolites.

**Table 3:** Characteristic differential metabolites in BH-PPG and NBH-PPG.

Grouping	Index	Differential metabolites	Metabolite categories	VIP	Log2FC	Type
BH-PPG/NBH-PPG VS NPG	MEDP878	N-methyl-L-glutamate	Amino acids and the metabolites	1.38	1.10	Up
	MEDP037	L-Asparagine acetic acid - L-phenylalanine acetic acid	Amino acids and the metabolites	1.08	1.37	Up
	MEDP575	Acadesine	Nucleotide and the metabolites	1.09	−1.52	Down
	MEDN736	2-(Methyl thiyl) ethanol	Alcohols	1.61	−1.19	Down
	MEDP362	Neopterin	Pteridine and the derivatives	1.34	−1.16	Down
	MEDN084	Benzoic acid	Benzene and the derivatives	1.39	−1.02	Down
	MEDN808	Inositol	Carbohydrate and the metabolites	1.53	−1.02	Down

BH-PPG VS NBH-PPG	MEDN698	1-Naphthol	Phenols and the derivatives	1.07	3.2	Up
	MEDP889	Cortisol	Lipid	1.85	2.57	Up
	MEDP171	Inosine	Nucleotide and the metabolites	1.06	1.44	Up
	MEDN751	(±) 12-Hydroxy-5Z, 8Z, 10E, 14Z-eicosapentaenoic acid	Oxidized lipid	1.15	1.34	Up
	MEDN286	3,4,5-Trimethoxy cinnamic acid	Organic acids and the derivatives	1.81	−1.90	Down
	MEDP118	4-Pyrazole compound acid	Pyridine and the derivatives	1.69	−1.34	Down
	MEDN334	Mandelic acid	Organic acids and the derivatives	2.38	−1.04	Down
	MEDN097	p-Hydroxyphenylacetic acid	Benzene and the derivatives	2.24	−1.01	Down

*Note.* The upper part of the table presents the significantly differential metabolites of BH-PPG and NBH-PPG compared to the normal control group. The lower part of the table presents the differential metabolites of BH-PPG compared to NBH-PPG.

## Data Availability

All data are included in the article are also available upon request to the authors.
